The article "Barriers to initiation of antiretroviral treatment in rural and urban areas of Zambia: a cross-sectional study of cost, stigma, and perceptions about ART" was published in 2010. Journal: J Int AIDS Soc.

# Barriers to initiation of antiretroviral treatment in rural and urban areas of Zambia: a cross-sectional study of cost, stigma, and perceptions about ART

**DOI:** 10.1186/1758-2652-13-8

**Published:** 2010-03-06

**Authors:** Matthew P Fox, Arthur Mazimba, Phil Seidenberg, Denise Crooks, Bornwell Sikateyo, Sydney Rosen

**Affiliations:** 1 Center for Global Health and Development, Boston University, Boston, MA, USA; 2 Boston University Center for International Health and Development - Zambia, Lusaka, Zambia; 3 Department of International Health, Boston University School of Public Health, Boston, MA, USA; 4 Ministry of Health, Lusaka, Zambia

## Abstract

**Background:**

While the number of HIV-positive patients on antiretroviral therapy (ART) in resource-limited settings has increased dramatically, some patients eligible for treatment do not initiate ART even when it is available to them. Understanding why patients opt out of care, or are unable to opt in, is important to achieving the goal of universal access.

**Methods:**

We conducted a cross-sectional survey among 400 patients on ART (those who were able to access care) and 400 patients accessing home-based care (HBC), but who had not initiated ART (either they were not able to, or chose not to, access care) in two rural and two urban sites in Zambia to identify barriers to and facilitators of ART uptake.

**Results:**

HBC patients were 50% more likely to report that it would be very difficult to get to the ART clinic than those on ART (RR: 1.48; 95% CI: 1.21-1.82). Stigma was common in all areas, with 54% of HBC patients, but only 15% of ART patients, being afraid to go to the clinic (RR: 3.61; 95% CI: 3.12-4.18). Cost barriers differed by location: urban HBC patients were three times more likely to report needing to pay to travel to the clinic than those on ART (RR: 2.84; 95% CI: 2.02-3.98) and 10 times more likely to believe they would need to pay a fee at the clinic (RR: 9.50; 95% CI: 2.24-40.3). In rural areas, HBC subjects were more likely to report needing to pay non-transport costs to attend the clinic than those on ART (RR: 4.52; 95% CI: 1.91-10.7). HBC patients were twice as likely as ART patients to report not having enough food to take ART being a concern (27% vs. 13%, RR: 2.03; 95% CI: 1.71-2.41), regardless of location and gender.

**Conclusions:**

Patients in home-based care for HIV/AIDS who never initiated ART perceived greater financial and logistical barriers to seeking HIV care and had more negative perceptions about the benefits of the treatment. Future efforts to expand access to antiretroviral care should consider ways to reduce these barriers in order to encourage more of those medically eligible for antiretrovirals to initiate care.

The article "Barriers to initiation of antiretroviral treatment in rural and urban areas of Zambia: a cross-sectional study of cost, stigma, and perceptions about ART" was published in 2010. Journal: J Int AIDS Soc.

## Background

It has been estimated that globally about 4 million HIV-positive people were on antiretroviral therapy (ART) at the end of 2008 [1]. In resource-limited settings, the number on treatment has increased dramatically since the large-scale roll out of ART. Despite the ever-increasing availability of ART in these settings, however, some patients eligible for treatment do not initiate ART even when it is available to them.

In Zambia, where national adult HIV prevalence is estimated at 14% to 16% [2,3], only between 50% and 66% of those in need of ART were accessing it as of 2007 [4,5]. Some of those who are not in care have deliberately opted not to seek it, while others lack the resources, information or motivation required to do so. Understanding why patients opt out of care, or are unable to opt in, is important to achieving the goal of universal access. Currently, little is known about what inhibits uptake of antiretroviral (ARV) treatment even when it is available to them.

The majority of research on barriers to accessing ART has been conducted in resource-rich environments [6-12], and has identified poverty, fear of side effects [7,9], lack of belief in the need for treatment [8], and fear of stigma [10] as important barriers. In resource-limited settings, where barriers to accessing care likely differ [13], far less research has been conducted. Reasons for not seeking available care in resource-limited settings are likely related to the cost of seeking treatment [14-16], the time and distance needed to travel to access care [17], stigma [14], fear of violence [18,19], and reliance on traditional medicine [20].

While some research has been conducted to identify these barriers, we have found no published quantitative studies in developing countries that have compared actual and perceived barriers to accessing ART between those who chose to initiate treatment and successfully accessed care and those who did not. This lack of a comparison makes it difficult to identify which factors have the strongest influence on treatment seeking and could be targeted to improve uptake. To understand why HIV-positive people who are medically eligible for ART do not initiate treatment, we surveyed patients on ART and patients believed to be accessing home-based care for HIV/AIDS, but who had not initiated ART, to identify barriers to and facilitators of ART uptake in rural and urban areas of Zambia.

## Methods

### Study sites

The study sites were HIV clinics and the surrounding catchment areas. Two sites were located in Zambia's Southern Province, one in an urban area in Livingstone (Maramba clinic), and one in a rural part of Choma District (Pemba clinic). A third site was urban and located in Lusaka (Chawama clinic) in Lusaka Province, and the fourth was in a rural part of Central Province in Chibombo (Chipembi Mission Clinic). All the sites, except Chipembi, were government clinics.

The article "Barriers to initiation of antiretroviral treatment in rural and urban areas of Zambia: a cross-sectional study of cost, stigma, and perceptions about ART" was published in 2010. Journal: J Int AIDS Soc.

The HIV prevalence in the study areas ranged from 14% in Southern Province to as high as 21% in Lusaka [2]. HIV treatment providers serving the sites were vastly different in size, but all were government clinics offering ART, prevention of mother to child transmission services, and voluntary counselling and testing. The rural sites each had between 400 and 600 active patients on ART, while the urban sites had between 2000 and 8000 patients on ART.

Within the catchment area of each study site clinic, we identified a home-based care programme that was providing services to patients who have terminal conditions, including confirmed and suspected HIV-positive patients who chose not to initiate ART. Home-based care (HBC) is provided by faith-based and other non-governmental organizations (NGOs) in Zambia; it offers palliative care to people in advanced stages of HIV. Three of the HBC groups were operating under the government clinic, while the fourth was NGO run.

### Study design and population

We conducted a cross-sectional survey by administering a questionnaire among confirmed and suspected HIV-positive adults (≥ 18 years old) believed to be medically eligible for ART (i.e., with CD4 counts of <200 cells/mm^3 ^or WHO stage III/IV [21]) at two rural and two urban sites in Zambia. Eligible subjects were those living within the catchment area of the ART clinic and were eligible for ART. To be able to identify barriers to seeking ART, we enrolled two groups of subjects: (1) clients of one or more home-based AIDS care programmes; and (2) patients on ART at the HIV clinics serving the same populations as the HBC programmes.

Our primary focus was on patients who were eligible for ART, but who chose not to initiate HIV treatment. Individuals who choose not to initiate ART are difficult to access as they do not present at a facility for HIV care. One way to identify HIV-infected people not on ART is through home-based care organizations, which care for patients in the community as they become ill. HBC programmes encourage eligible subjects to initiate ART, but also provide palliative care for those who decline. Thus, by working with HBC programmes to enrol HBC patients, we were able to select a sample of ill patients who had chosen not to initiate ART.

Subjects in the HBC group comprised individuals believed by HBC caregivers to be medically eligible for ARV treatment, but not actively on treatment. We excluded all HBC subjects who were on ART, as well as subjects who had received ARVs prior to study enrolment. Because this population is difficult to identify and because we wished to respect patients' decisions and attitudes towards treatment, we relied on HBC caregivers to identify eligible subjects. It is possible that some of these subjects were using HBC services for non-HIV-related conditions as an HIV diagnosis is not required for HBC care. However, we asked HBC staff to refer to our study only those patients who had been screened for ART eligibility using WHO staging.

The article "Barriers to initiation of antiretroviral treatment in rural and urban areas of Zambia: a cross-sectional study of cost, stigma, and perceptions about ART" was published in 2010. Journal: J Int AIDS Soc.

Comparison subjects are those actively on ART and represent the population able to access ARV treatment. For comparability, we enrolled subjects receiving HIV care from the clinic serving the same catchment areas as those of the HBC programmes. We limited this population to subjects on ART for at least three months because there is a relatively high attrition from ARV programmes in the first three months, and subjects who did not remain on ART beyond three months would not be an appropriate group to represent those who were able to access care [22]. We further limited the comparison population to those on ART for less than six months to maximize their ability to recall events at the time of the decision to begin treatment.

### Data collection

HBC subjects were interviewed at home by a trained interviewer accompanied by an HBC caregiver. Any subject in the HBC group who expressed an interest in initiating HIV treatment was referred to the local HIV clinic with assistance from the HBC programme. ARV subjects were screened for eligibility by clinic nurses from the list of all registered patients and selected with n^th ^name sampling. Eligible subjects willing to be interviewed were referred to a trained interviewer, who conducted the interview during a routine clinic visit.

Questions were phrased differently for those in the HBC group and those in the ARV group. Typically, HBC subjects were asked hypothetical questions, while ARV subjects were asked about their actual experience. For example, ARV subjects were asked about the transportation they actually took to the HIV clinic or what concerns they had about taking ART, while HBC subjects were asked about what transportation they thought they would use to get to the HIV clinic or what concerns people have about taking ART.

All subjects gave verbal consent to be interviewed. The study was approved by the Boston University Institutional Review Board and the University of Zambia Research Ethics Committee.

### Analytic variables and statistical analysis

We asked subjects about transportation to the clinic (mode, time and costs) and their concerns about ART at the time they were considering initiating ART. Subjects in the HBC group who had never actively decided to forgo ART were asked about their current concerns. Concerns were categorized as being about: (1) fear/stigma; (2) perceived benefits of ARVs; (3) harms of and/or difficulties with ARVs; (4) need for ARVs; and (5) barriers to accessing ARVs. We present the results as simple percentages and relative risks (RR) and corresponding 95% confidence intervals (CI). To look for differences in barriers to care seeking by site, we stratified our analyses by location (rural or urban). Where strong differences were found, we also analyzed data stratified by gender (data not shown).

The article "Barriers to initiation of antiretroviral treatment in rural and urban areas of Zambia: a cross-sectional study of cost, stigma, and perceptions about ART" was published in 2010. Journal: J Int AIDS Soc.

## Results

### Socio-economic and demographic characteristics

We surveyed 800 subjects evenly distributed between study sites and between subjects on ART and those in home-based care (Table 1). About two in three subjects were female and more than half were between 20 and 39 years of age, similar to the distribution of all patients on ART in Zambia.

**Table 1:** Demographic characteristics of subjects in a cross-sectional survey in rural and urban areas of Zambia*

Demographic characteristics	Urban: n (%)		Rural: n (%)	
	
	ARVs (N = 200)	HBC (N = 200)	ARVs (N = 200)	HBC (N = 200)
**Female**	129 (65)	122 (61)	133 (67)	121 (61)
**Age**				
<30	52 (26)	52 (26)	33 (16)	29 (15)
30.0 - 39.9	89 (45)	68 (34)	83 (42)	85 (42)
40.0 - 49.9	44 (22)	30 (15)	72 (36)	47 (23)
50.0 - 59.9	12 (6)	32 (16)	8 (4)	18 (9)
60.0+	3 (2)	18 (9)	2 (1)	18 (9)
Missing	0 (0)	0 (0)	2 (1)	3 (2)
**Marital status**				
Single	31 (16)	28 (14)	25 (13)	28 (14)
Engaged/married	110 (55)	94 (47)	106 (53)	126 (63)
Widowed/divorced/separated	59 (30)	78 (39)	69 (35)	46 (23)
**Common language used**				
Nyanja	59 (30)	65 (33)	21 (11)	18 (9)
Bemba	44 (22)	29 (15)	20 (10)	12 (6)
Tonga	28 (14)	37 (18)	101 (51)	103 (51)
Lozi	41 (21)	33 (17)	15 (8)	10 (5)
Others	28 (14)	36 (17)	43 (22)	57 (28)
**Educational level**				
Never attended school	11 (6)	18 (9)	10 (5)	22 (11)
Attended/completed primary school	84 (42)	87 (44)	99 (50)	127 (64)
Attended secondary school	59 (29)	71 (35)	69 (34)	40 (20)
Completed secondary school	36 (18)	23 (11)	18 (9)	6 (3)
Attended/completed tertiary education	10 (5)	1 (1)	4 (2)	5 (2)
**Ability to communicate in English**				
Very well	58 (29)	27 (14)	23 (12)	18 (9)
Somewhat	73 (36)	88 (43)	104 (52)	69 (34)
Not able to	68 (34)	85 (43)	73 (37)	113 (57)
Missing	1 (1)	0 (0)	0 (0)	0 (0)
**Respondents' most important economic activity**				
Formal employment	26 (13)	19 (9)	26 (13)	25 (12)
Self-employed	95 (47)	85 (42)	114 (57)	105 (52)
Unemployed	71 (36)	77 (39)	47 (24)	53 (27)
Other	8 (4)	19 (10)	13 (6)	16 (8)
Missing	0 (0)	0 (0)	0 (0)	1 (1)
**Self-reported economic status**				
Much or somewhat poorer than most	97 (48)	133 (66)	108 (54)	124 (62)
About the same as most	84 (42)	61 (30)	68 (34)	57 (28)
Somewhat or much wealthier than most	18 (9)	5 (2)	24 (12)	18 (9)
Missing	1 (1)	1 (1)	0 (0)	1 (1)
**Health-seeking decisions made primarily by:**				
Self	100 (50)	96 (48)	114 (57)	127 (63)
Parents	32 (16)	25 (13)	31 (15)	17 (9)
Spouse	31 (16)	24 (12)	36 (18)	43 (21)
Others	37 (18)	55 (27)	19 (10)	12 (6)
Missing	0 (0)	0 (0)	0 (0)	1 (1)
**Primary source of money for buying household food**				
Respondent (self)	110 (55)	102 (51)	125 (62)	127 (63)
Parents	17 (8)	13 (6)	25 (13)	5 (2)
Spouse	46 (23)	35 (18)	39 (20)	58 (29)
Other	27 (14)	50 (25)	11 (5)	9 (5)
Missing	0 (0)	0 (0)	0 (0)	1 (1)
**Frequency of going without a meal**				
Usually/always	54 (27)	14 (7)	28 (14)	31 (15)
Sometimes	114 (57)	133 (66)	109 (55)	92 (46)
Seldom/almost never	32 (16)	53 (27)	63 (32)	76 (38)
Missing	0 (0)	0 (0)	0 (0)	1 (1)
**Household source of drinking water**				
Tap inside the house	13 (7)	5 (2)	2 (1)	6 (3)
Own tap outside the house	73 (37)	70 (35)	8 (4)	12 (6)
Shared community source	111 (56)	124 (62)	186 (94)	176 (88)
Other	3 (2)	1 (0)	4 (2)	5 (2)
Missing	0 (0)	0 (0)	0 (0)	1 (1)
**Type of sanitary facility**				
Flush toilet	64 (32)	37 (18)	5 (3)	4 (2)
Traditional pit latrine	111 (56)	116 (58)	161 (81)	114 (57)
Ventilated improved pit latrine	12 (6)	22 (11)	3 (2)	0 (0)
None	13 (7)	25 (13)	31 (16)	80 (40)
Missing	0 (0)	0 (0)	0 (0)	2 (1)
**Households reported to have or own**				
Electricity	97 (49)	47 (24)	10 (5)	11(5)
Cellular phone	144 (72)	99 (50)	79 (40)	56 (28)
Radio	135 (68)	94 (47)	125 (63)	96 (48)
Television	115 (58)	77 (39)	24 (12)	30 (15)

Those interviewed were generally of low socio-economic status. Access to flush toilets was reported by <14% of subjects and was very rare in rural areas (2.3%). Between 25% and 40% of all subjects reported themselves to be unemployed, and about 60% said they were much or somewhat poorer than most in their community. ART subjects were twice as likely as HBC subjects to have completed secondary school or higher (23% vs. 12% in urban areas, 11% vs. 5% in rural areas).

The article "Barriers to initiation of antiretroviral treatment in rural and urban areas of Zambia: a cross-sectional study of cost, stigma, and perceptions about ART" was published in 2010. Journal: J Int AIDS Soc.

We found that subjects in urban areas were more likely to report being able to speak English well and report a high level of education compared with rural areas. Females were more likely to be in the 20-29 age range than males (23.6% vs. 13.9%, respectively) and to be widowed than men (25.3% vs. 10.9%, respectively) They were also less likely to have completed secondary school or higher (8.9% vs. 19.7%, respectively), speak English well (11.9% vs. 22.5%, respectively), or be the main provider of food in the household (45.2% vs. 80.0%, respectively). The differences persisted even when stratified by study group (ART vs. HBC).

### Transportation, cost of seeking treatment

Table 2 shows differences between the study groups in terms of transportation to the clinic, costs of seeking treatment, and perceptions of care at the HIV clinic by rural/urban status. While only 16% of subjects overall reported that it would be very difficult for them to get to an ART clinic, HBC subjects were 50% more likely to report this difficulty than those on ART (RR: 1.48; 95% CI: 1.07-2.05).

**Table 2:** Transportation to the clinic, cost of seeking treatment and perceptions of care at the HIV*

	Urban			Rural			Total
**Exposure**	**Home-based care**	**On ART**	**Relative risk** **(95% CI)**	**Home-based care**	**On ART**	**Relative risk** **(95% CI)**	**Relative risk** **(95% CI)**
**Transport used (would be used) to get to the HIV clinic**							
Walked	193/200 (96.5%)	180/200 (90.0%)	1.07 (1.02 - 1.13)	188/200 (94.0%)	143/200 (71.5%)	1.31 (1.20 - 1.44)	1.18 (1.12 - 1.24)
Taxi	13/200 (6.5%)	27/200 (13.5%)	0.48 (0.26 - 0.91)	7/200 (3.5%)	6/200 (3.0%)	1.17 (0.40 - 3.41)	0.61 (0.35 - 1.04)
Private car	2/200 (1.0%)	7/200 (3.5%)	0.29 (0.06 - 1.36)	14/200 (7.0%)	11/200 (5.5%)	1.27 (0.59 - 2.74)	0.89 (0.46 - 1.72)
Bicycle	2/200 (1.0%)	2/200 (1.0%)	1.00 (0.14 - 7.03)	21/200 (10.5%)	49/200 (24.5%)	0.43 (0.27 - 0.69)	0.45 (0.28 - 0.72)
Bus	18/200 (9.0%)	22/200 (11.0%)	0.82 (0.45 - 1.48)	1/200 (0.5%)	18/200 (9.0%)	0.06 (0.01 - 0.41)	0.48 (0.28 - 0.81)
**Barriers to seeking care**							
It is very difficult to get to the clinic	34/200 (17.0%)	21/200 (10.5%)	1.62 (0.97 - 2.69)	43/199 (21.6%)	31/200 (15.5%)	*1.39 (0.92 - 2.12)*	1.48 (1.07 - 2.05)
I can't leave my work to go to the ARV clinic	25/181 (13.8%)	17/195 (8.7%)	1.58 (0.89 - 2.84)	12/174 (6.9%)	5/191 (2.6%)	2.63 (0.95 - 7.33)	1.83 (1.10 - 3.04)
I do not have time to go to the ARV clinic	2/197 (1.0%)	0/198 (0%)		9/196 (4.6%)	4/200 (2.0%)	2.30 (0.72 - 7.33)	2.78 (1.55 - 4.99)
The ARV clinic is too far for me to travel to	52/190 (27.4%)	16/197 (8.1%)	3.37 (2.00 - 5.69)	81/196 (41.3%)	55/198 (27.8%)	1.49 (1.12 - 1.97)	1.92 (1.64 - 2.24)
**To visit the clinic, I have to/would have to:**							
Pay a fee at the clinic	19/200 (9.5%)	2/200 (1.0%)	9.50 (2.24 - 40.3)	9/199 (4.5%)	11/200 (5.5%)	0.82 (0.35 - 1.94)	2.16 (1.14 - 4.11)
Pay to travel	96/199 (48.2%)	34/200 (17.0%)	2.84 (2.02 - 3.98)	29/197 (14.7%)	37/200 (18.5%)	0.80 (0.51 - 1.24)	1.78 (1.38 - 2.30)
Spend night away from home	1/149 (0.7%)	2/127 (1.6%)	0.43 (0.04 - 4.65)	4/198 (2.0%)	2/199 (1.0%)	2.01 (0.37 - 10.9)	1.17 (0.32 - 4.34)
Pay someone to take over my tasks	27/200 (13.5%)	11/200 (5.5%)	2.45 (1.25 - 4.81)	5/198 (2.5%)	3/200 (1.5%)	1.68 (0.41 - 6.95)	2.30 (1.25 - 4.24)
Other costs	24/200 (12.0%)	22/199 (11.1%)	1.09 (0.63 - 1.87)	27/199 (13.6%)	6/200 (3.0%)	4.52 (1.91 - 10.7)	1.82 (1.17 - 2.83)
Visit the clinic > once/month	34/109 (31.2%)	10/199 (5.0%)	6.21 (3.19 - 12.1)	40/152 (26.3%)	21/199 (10.6%)	2.49 (1.54 - 4.05)	3.64 (2.47 - 5.37)
**Do you perceive the ___ at the clinic to be good/excellent?**							
Service	81/200 (40.5%)	131/200 (65.5%)	0.62 (0.51 - 0.75)	117/199 (58.8%)	170/200 (85.0%)	0.69 (0.61 - 0.79)	0.66 (0.59 - 0.74)
Provider time	91/200 (45.5%)	139/198 (70.2%)	0.65 (0.54 - 0.77)	87/199 (43.7%)	150/200 (75.0%)	0.58 (0.49 - 0.70)	0.61 (0.54 - 0.70)
Waiting time	35/199 (17.6%)	43/199 (21.6%)	0.81 (0.55 - 1.22)	42/198 (21.2%)	45/200 (22.5%)	0.94 (0.65 - 1.37)	0.88 (0.67 - 1.15)
Counselling	112/200 (56.0%)	147/199 (73.9%)	0.76 (0.65 - 0.88)	108/199 (54.3%)	147/200 (73.5%)	0.74 (0.63 - 0.86)	0.75 (0.67 - 0.83)
Staff concern	74/200 (37.0%)	123/199 (61.8%)	0.60 (0.48 - 0.74)	81/198 (40.9%)	148/200 (74.0%)	0.55 (0.46 - 0.67)	0.57 (0.50 - 0.66)
Convenience of clinic hours	154/200 (77.0%)	136/199 (68.3%)	1.13 (1.00 - 1.27)	119/199 (59.8%)	132/199 (66.3%)	0.90 (0.78 - 1.05)	1.02 (0.92 - 1.12)

When asked to describe the transport they use (or would use) to get to the HIV clinic, all forms of transport other than walking (taxi, private car, bicycle and bus) were less frequently mentioned by HBC subjects, though this differed by location. All forms of transport other than walking were reported by <15% of the population, except for bicycles in the rural areas.

The article "Barriers to initiation of antiretroviral treatment in rural and urban areas of Zambia: a cross-sectional study of cost, stigma, and perceptions about ART" was published in 2010. Journal: J Int AIDS Soc.

Overall, HBC participants were 40% to 55% less likely to take a taxi (0.61; 95% CI: 0.35-1.04), a bicycle (RR: 0.45; 95% CI: 0.28-0.72) or a bus (RR: 0.48; 95% CI: 0.28-0.81) as part of their journeys, but these differed by location. In rural areas, HBC patients were much less likely to report that they would use a bicycle (10.5% vs. 24.5%, RR: 0.43; 95% CI: 0.27-0.69) or a bus (0.5% vs. 9.0%, RR: 0.06; 95% CI: 0.01-0.41) than those in the ART group, but only minor differences were observed in these modes in the urban areas. In urban areas, HBC patients were much less likely to report they would use a taxi (6.5% vs. 13.5%, RR: 0.48; 95% CI: 0.26-0.91) than those in the ART group.

Cost barriers for HBC patients also differed by location. About 25% of all subjects reported that they would need to pay a fee to travel to a clinic, but in urban areas, HBC subjects were nearly three times more likely to report believing this than those on ART (RR: 2.84; 95% CI: 2.02-3.98), with no difference in the rural areas. This effect was almost entirely among men (male HBC vs. ART patients: RR 14.1; 95% CI: 1.89-105; females 1.08; 95% CI: 0.50-2.36). In rural areas, HBC patients were more likely to report needing to pay costs other than transport and clinic fees than those on ART (13.6% vs. 3.0%, RR: 4.52; 95% CI: 1.91-10.7). These patients answered yes to the question, "Are there any other costs that you must pay to obtain treatment for HIV/AIDS, either in money, time, lost income, or anything else, that have not been mentioned yet?".

The article "Barriers to initiation of antiretroviral treatment in rural and urban areas of Zambia: a cross-sectional study of cost, stigma, and perceptions about ART" was published in 2010. Journal: J Int AIDS Soc.

Most of this association was among women (male HBC vs. ART patients: 1.18; 95% CI: 0.51-2.71; female HBC vs. ART patients: 4.33; 95% CI: 1.65-11.4). HBC subjects were not more likely to report needing to spend a night away from home than those on ART (1.4% vs. 1.2%), regardless of location, suggesting that while those on ART might live closer to the clinic, the differences were not so great that the journey could not be completed in a day.

While very uncommon overall (5%), in urban areas, HBC participants were twice as likely to report believing that they would have to pay a fee at the clinic than those on ART (RR: 9.50; 95% CI: 2.24-40.3) and that they would have to pay someone to take over their tasks to attend the clinic (RR: 2.45; 95% CI: 1.25 - 4.81). Nearly 30% of those in the HBC programme reported believing that they would need to attend the clinic more than once per month, nearly three times more than those on ART in rural areas (RR: 2.49; 95% CI: 1.54-4.05) and roughly six times more than those on ART in urban areas (RR: 6.21; 95% CI: 2.47-5.37). While about 10% of HBC subjects reported that they could not leave work to seek ARVs, this was substantially more than ARV recipients in both rural and urban areas (RR: 1.83; 95% CI: 1.10-3.04).

### Perceptions about care and ARVs

In response to questions about subjects' perceptions of the ART clinic services, HBC subjects reported less favourable impressions than those who had actually experienced the care (Table 2), with little variation by location or gender. Nearly 70% of subjects in both groups felt the convenience of the clinic was good or excellent, and about 20% in both groups felt the waiting times were good or excellent. However, on all other indicators (including service, provider time, counselling and staff concern), HBC subjects perceived the services to be worse than did ART subjects.

Fear of attending the clinic was very common (Table 3) in all locations, with more HBC subjects than ART subjects reporting being afraid to go to the clinic (RR: 3.61; 95% CI: 2.80-4.66) and that if they went to the clinic, people would not like them (RR: 2.28; 95% CI: 1.82-2.87). Concerns about fear and stigma were also relatively common (Table 3), with 20% to 30% of all participants reporting some concern about stigma, but were much more common among HBC participants.

The article "Barriers to initiation of antiretroviral treatment in rural and urban areas of Zambia: a cross-sectional study of cost, stigma, and perceptions about ART" was published in 2010. Journal: J Int AIDS Soc.

**Table 3:** Concerns about taking antiretroviral therapy in a cross-sectional survey in Zambia*

	Urban			Rural			Total
At the time of making the decision about taking ARVs (or in general*), I (people) believe(d) that...	**Home-based care**	**On ART**	**Relative risk** **(95% CI)**	**Home-based care**	**On ART**	**Relative risk** **(95% CI)**	**Relative risk** **(95% CI)**

**Benefits of ARVs**							
If I take ARVs...							
I will feel better/stop being sick	154/199 (77.4%)	164/197 (83.2%)	0.93 (0.84 - 1.03)	134/199 (67.3%)	122/200 (61.0%)	1.10 (0.95 - 1.28)	1.00 (0.92 - 1.09)
I will be happier	29/199 (14.6%)	40/198 (20.2%)	0.72 (0.47 - 1.12)	21/198 (10.6%)	17/200 (8.5%)	1.25 (0.68 - 2.29)	0.88 (0.62 - 1.25)
I will be able to take care of my family	43/199 (21.6%)	62/198 (31.3%)	0.69 (0.49 - 0.97)	44/199 (22.1%)	40/199 (20.1%)	1.10 (0.75 - 1.61)	0.85 (0.66 - 1.09)
If I do not take ARV treatment I will die	151/190 (79.5%)	164/194 (84.5%)	0.94 (0.86 - 1.03)	157/187 (84.0%)	155/198 (78.3%)	1.07 (0.97 - 1.18)	1.00 (0.94 - 1.07)
**Fear and stigma**							
I am afraid of stigma	61/198 (30.8%)	31/197 (15.7%)	1.96 (1.33 - 2.88)	88/199 (44.2%)	50/198 (25.3%)	1.75 (1.32 - 2.33)	1.83 (1.45 - 2.31)
I am afraid of abuse	37/198 (18.7%)	18/198 (9.1%)	2.06 (1.21 - 3.48)	54/199 (27.1%)	37/199 (18.6%)	1.46 (1.01 - 2.11)	1.65 (1.22 - 2.24)
If I go to the clinic people will not like me	88/193 (45.6%)	38/187 (20.3%)	2.24 (1.62 - 3.10)	86/188 (45.7%)	38/193 (19.7%)	2.32 (1.68 - 3.21)	2.28 (1.82 - 2.87)
I am afraid to go to the ARV clinic	100/185 (54.1%)	32/195 (16.4%)	3.29 (2.34 - 4.64)	99/185 (53.5%)	26/194 (13.4%)	3.99 (2.72 - 5.85)	3.61 (2.80 - 4.66)
My family doesn't want me to take ARVs	2/197 (1.0%)	0/198 (0%)		19/198 (9.6%)	5/200 (2.5%)	3.84 (1.46 - 10.1)	4.23 (1.61 - 11.1)
**Harms of/difficulties with ARVs**							
ARVs will make me sick	47/197 (23.9%)	25/198 (12.6%)	1.89 (1.21 - 2.94)	40/199 (20.1%)	35/200 (17.5%)	1.15 (0.76 - 1.73)	1.46 (1.08 - 1.96)
I do not have enough food to take ARVs	50/198 (25.3%)	19/198 (9.6%)	2.63 (1.61 - 4.30)	57/198 (28.8%)	34/200 (17.0%)	1.69 (1.16 - 2.47)	2.03 (1.51 - 2.73)
ARVs are bad	28/174 (16.1%)	21/189 (11.1%)	1.45 (0.86 - 2.45)	30/184 (16.3%)	14/198 (7.1%)	2.31 (1.26 - 4.21)	1.79 (1.21 - 2.66)
If I take ARV treatment I will die	62/187 (33.2%)	20/185 (10.8%)	3.07 (1.93 - 4.86)	81/189 (42.9%)	29/199 (14.6%)	2.94 (2.02 - 4.28)	2.98 (2.23 - 3.99)
**Need for ARVs**							
I do not want to take any medicine	48/173 (27.7%)	15/198 (7.6%)	3.66 (2.13 - 6.30)	29/181 (16.0%)	9/197 (4.6%)	3.51 (1.71 - 7.21)	3.58 (2.32 - 5.53)
I do not need ARVs because I am not sick	5/62 (8.1%)	1/197 (0.5%)	15.9 (1.89 - 133)	1/52 (1.9%)	0/200 (0%)		20.89 (2.54 - 172)
I would rather take traditional medicines	15/177 (8.5%)	4/193 (2.1%)	4.09 (1.38 - 12.1)	21/176 (11.9%)	5/191 (2.6%)	4.56 (1.76 - 11.8)	4.35 (2.13 - 8.90)

* Those in the HBC programme who did not actively decide to forgo ART were asked if they currently believed each question, and questions were asked about concerns that "people" had about ARVs.

The article "Barriers to initiation of antiretroviral treatment in rural and urban areas of Zambia: a cross-sectional study of cost, stigma, and perceptions about ART" was published in 2010. Journal: J Int AIDS Soc.

About 5% of HBC subjects reported that a family member did not want them to take ARVs, but in the rural areas, substantially more HBC subjects reported this concern than ARV subjects in the rural areas (9.6% vs. 2.5%; RR: 3.84; 95 CI: 1.46-10.1). In most cases, reports of stigma comparing male HBC patients and male ART patients showed similar associations to those comparing female HBC patients and female ART patients. The one important exception to this was that we observed a somewhat greater association between being in the HBC group versus the ART group in terms of reported fear of abuse when we compared only females (RR female HBC vs. female ART: 1.82; 95% CI: 1.27-2.61) versus when we compared only males (RR male HBC vs. male ART: 1.40; 95% CI: 0.80-2.45).

Most subjects, regardless of study group, identified benefits of ARVs (Table 3). Both groups were equally likely to report that ART would make them feel better (a common belief) and that they would be happier if they took ART. In urban areas, however, the HBC group was somewhat less likely to report they would be better able to take care of their families if they took ART compared with the urban ART group (RR: 0.69; 95% CI: 0.49-0.97).

HBC subjects were much more likely than ART subjects to report concerns about the harms of or difficulties with ARVs. In particular, 27% of HBC subjects, but only 13% of ART subjects, reported not having enough food to take ARVs being a concern for initiating ART (RR: 2.03; 95% CI: 1.51-2.73), with similar associations being observed in both rural and urban areas. While 13% of ART subjects reported believing that they would die if they took ARVs when they were making the decision whether or not to initiate ART, 38% of HBC subjects reported this concern (RR: 2.98; 95% CI: 2.23-3.99). The association was stronger for males comparing HBC patients and ART patients (RR: 4.03; 95% CI: 2.25-7.21) than for females (RR: 2.66; 95% CI: 1.89-3.72).

HBC subjects were much more likely to report feeling they did not need ARVs because they were not sick than those on ARVs (5.3% vs. 0.3% respectively), although it was uncommon overall and was observed almost entirely in the urban areas. In urban areas, HBC subjects were also more likely than those on ART to report that ARVs would make them sick (RR: 1.89; 95% CI: 1.21-2.94). While only 2.3% of ARV subjects reported a preference for traditional medicines over ARVs at the time of making their decision to initiate ART, 10.2% of HBC participants reported this preference (RR: 4.35; 95% CI: 2.12-8.90), with hardly any differences by location.

The article "Barriers to initiation of antiretroviral treatment in rural and urban areas of Zambia: a cross-sectional study of cost, stigma, and perceptions about ART" was published in 2010. Journal: J Int AIDS Soc.

## Discussion

In the early years of public treatment programmes in sub-Saharan Africa, numbers of new patients initiating ART grew exponentially, and demand exceeded the supply of treatment slots available. Rationing of treatment by providers was necessary, but eligible patients also rationed care implicitly through their decisions about whether, and when, to seek treatment. As clinic capacity continues to expand, patient self-selection into ART programmes will be become increasingly important in determining how close countries can come to the goal of universal access programmes. Reaching universal access will require increasing access to patients who currently are eligible for ART, but are either unable or unwilling to seek it. Designing effective interventions to reduce barriers to access requires that we understand these patients' reasons for avoiding treatment.

We interviewed 400 people who were presumed eligible as they were in palliative care for HIV/AIDS and had not initiated ARVs. This suggests that while HBC caregivers are able to recognize their illnesses, they are not able to get these patients into care. The most recent Zambian Demographic and Health Survey found that among adults aged 15 to 49, while 82% knew that a healthy person could be HIV positive, only 39% of women and 22% of men had ever tested for HIV [2]. Taken together, this suggests that while attitudes towards HIV may be changing as ART becomes more widely available, many still choose never to acknowledge their status, and referral systems designed to move people from knowledge of the problem to awareness of their own status and on to enrolment in care and treatment must be strengthened.

We found that HBC subjects perceived they would face greater costs to seeking ART, both in terms of direct payment for care and in the costs of travelling to the clinic and the opportunity costs of seeking care. This is similar to qualitative findings from Tanzania [14], Zambia [15] and Malawi [16]. A recent cross-sectional survey in Cameroon [23] found that those on ART were of higher socio-economic status than those eligible for ART but not on it.

While removing user fees has been shown to be effective at increasing adherence [24], these studies and our results suggest that efforts to get those who could benefit from ARVs into care will have to find ways to reduce the perceived and actual costs of accessing care beyond the removal of clinic fees.

The article "Barriers to initiation of antiretroviral treatment in rural and urban areas of Zambia: a cross-sectional study of cost, stigma, and perceptions about ART" was published in 2010. Journal: J Int AIDS Soc.

Interestingly, our study found differences in urban and rural setting in the types of financial barriers faced by those not on ART. Urban HBC patients were more likely to report believing that they would face transport and clinic cost barriers, while rural HBC patients perceived that they would face more non-transport cost barriers if they accessed care. This suggests that strategies like providing transport vouchers or using mobile clinics to deliver ARVs may be able to reduce these barriers. However, our findings make it clear that the barriers experienced in accessing ART in rural and urban areas differ, and that in order to effectively reduce barriers to care, interventions will need to be tailored to the specific needs of the population.

We found that HBC patients also had substantially greater negative perceptions about ART than those on ART, and these negative perceptions were common, regardless of the study site. Most subjects, regardless of which group they were in, recognized the survival benefits of ARVs, regardless of location. This suggests that efforts to educate the public about HIV/AIDS treatment have succeeded in conveying information. They have been less successful in overcoming actual and perceived barriers to action, however, as indicated by our survey.

Some misperceptions about ARVs were more common among the HBC population in our study and reports of stigma were common. More than 50% of HBC subjects said that they were afraid to go to the HIV clinic. We found no important differences in stigma across the rural and urban sites, regardless of the measure used. Stigma and fear of violence has been previously identified as a barrier to accessing care [14,18,19,25,26]. Our results suggest that even as access to care has become more common, stigma has not disappeared and continues to play a strong role in the decision-making process around ARVs.

Reports of concerns over stigma were common among all subjects in our study (nearly 30% of the total population mentioned that stigma had been experienced), but were more common among those in the HBC programme. In absolute terms, depending on the measure used, those in the HBC group had between 20% and 40% more subjects reporting stigma than those in the ART group. Two examples of this were: "I am afraid to go to the ARV clinic" (54% vs. 15%); and "If I go to the clinic people will not like me" (46% vs. 20%). Stigma was the single strongest predictor of not being in care in absolute terms, and this suggests that more work needs to be done to remove feelings of stigma in the community.

The article "Barriers to initiation of antiretroviral treatment in rural and urban areas of Zambia: a cross-sectional study of cost, stigma, and perceptions about ART" was published in 2010. Journal: J Int AIDS Soc.

Concern about needing additional food intake upon initiating ART has also previously been identified as a barrier to ART initiation [14,27,28]. We were able to quantify the increase compared with subjects on ART and found that HBC subjects were three times more likely to report concerns about not having enough food to take ARVs than those on ARVs. We found that this association between not being on ART and concerns about food held true in both rural and urban areas and among both men and women, suggesting that this may be a barrier experienced by many subpopulations of HIV-infected ART eligible patients.

We cannot tell from our data whether those in the HBC group were less able to access food or whether those on ART were better able to access food after initiating ART because they were able to return to work. However, provision of food to those in care could help increase a willingness to initiate care, although it would also increase costs, be difficult to sustain over time and may pose ethical issues in communities where food insecurity is common.

Our study had several strengths. We interviewed 800 subjects, which allowed us to conduct one of the largest and most comprehensive analyses of barriers to ART care that yet exists. We also included both rural and urban sites within Zambia, which helped improve the generalizability of our findings. Future efforts to determine how barriers and facilitators to accessing ARVs differ across rural and urban areas will help to further target interventions to reduce such barriers.

While our study was able to determine some key barriers to accessing care, it had several limitations. First, our target sample was not limited to subjects who were known to be HIV infected and eligible for ART, and who opted out of treatment. We felt it would be prohibitively difficult to identify these subjects and therefore chose a sample of HBC subjects believed by HBC caregivers to be eligible for, but not on, ART. Some subjects in this group may not have been eligible for ART, and it is also possible that HBC caregivers mistook some illnesses for HIV/AIDS.

It is not clear what impact this would have had on our findings, but we note that there was little difference in our results when the analysis was limited to subjects who told us they had actively made the decision not to initiate ART. In addition, patients in HBC care are likely to have had counselling about HIV and ART from the HBC caregivers. This would likely have the effect of making the two populations more similar with respect to their attitudes towards ART. Thus our findings should be interpreted as conservative estimates of the magnitude of the barriers to ART.

The article "Barriers to initiation of antiretroviral treatment in rural and urban areas of Zambia: a cross-sectional study of cost, stigma, and perceptions about ART" was published in 2010. Journal: J Int AIDS Soc.

Second, we relied on subject recall of their concerns about initiating ART. Using this approach, we could not tell the difference between actual and perceived barriers to care seeking. In addition, for those who had not actively made a decision to forgo ART, we had to ask about what those in their community felt were concerns about ART. Inevitably, some recall bias results when this approach is used. Those on ART, particularly those having a positive experience, would be less likely to report serious barriers to care seeking. While we could not remove this bias completely, we sought to mitigate it by asking subjects who had initiated ART to recall their concerns at the time they were making the decision whether or not to initiate care.

## Conclusions

In conclusion, we found that patients in home-based care for HIV/AIDS who never initiated ART experienced greater perceived financial and logistical barriers to seeking HIV care than those on ART. They were more likely to identify concerns about needing food if they initiated ART, costs for transportation and care, negative attitudes towards ARVs, and stigma as common concerns about seeking treatment. Future efforts to expand access to ARV care should consider ways to reduce these barriers in order to encourage more of those medically eligible for ARVs to initiate care.

## Competing interests

The authors declare that they have no competing interests.

## Authors' contributions

MF contributed to the design of the study, analyzed the data, and wrote the first draft of the manuscript. AM contributed to the design of the study, assisted in analyzing and interpreting the data, and contributed to editing the manuscript. PS assisted in analyzing and interpreting the data, and contributed to editing the manuscript. DC oversaw data collection, assisted in interpreting the data, and contributed to editing the manuscript. BS contributed to interpreting the data and to the final manuscript. SR contributed to the design of the study and the interpretation of the data, and contributed to writing the first manuscript. All authors have given final approval for the manuscript.
